The article "Clinical Outcomes of Repair of Complete Detachment of Medial Collateral Ligament at the Tibial Insertion in Bilateral Total Knee Arthroplasty" was published in 2022. Journal: Evid Based Complement Alternat Med.

# Clinical Outcomes of Repair of Complete Detachment of Medial Collateral Ligament at the Tibial Insertion in Bilateral Total Knee Arthroplasty

**DOI:** 10.1155/2022/7266233

**Published:** 2022-07-21

**Authors:** Cheng Jin, Eun-Kyoo Song, Quan-He Jin, Jong-Keun Seon, Si-Mei Sun

**Affiliations:** ^1^Zhoushan Hospital, Zhejiang University School of Medicine, Zhoushan, China; ^2^Center for Joint Disease, Chonnam National University Hwasun Hospital, Hwasun, Republic of Korea; ^3^Department of Orthopaedic Surgery, Affiliated Sir Run Run Hospital of Nanjing Medical University, Nanjing 211166, China

## Abstract

**Purpose:**

Complete detachment of the medial collateral ligament (MCL) may occur during medial release of total knee arthroplasty (TKA) in patients with severe varus knee osteoarthritis. This study was to determine functional and stability outcomes of repaired knee with complete detachment of MCL compared to those of contralateral nondetached MCL in patients with bilateral TKA.

**Methods:**

Records of 1052 consecutive knees undergoing bilateral TKA from 2003 to 2015 were retrospectively reviewed. Of which, 45 patients were repaired for complete MCL detachment injury (2.1%) at tibial insertion in one side (repaired group). MCL was not detached in the contralateral side (control group). Clinical evaluation was performed preoperatively and at the final follow-up using KS and WOMAC scores between two groups. Similarly, stability was compared on a valgus stress radiograph between two groups.

**Results:**

Two patients had insufficient data. Hence, 43 patients were included after a minimum of 5 years follow-up. There were no significant differences in terms of alignment and clinical outcomes between the two groups either preoperatively or at the final follow-up (*p* > 0.05). Radiographic stability also showed no differences between repaired and control groups in extension and 30° of flexion (*p*=0.208 and *p*=0.125).

**Conclusions:**

For tibial detachment of the MCL during TKA, repair with suture anchor provided good clinical and stability results, similar to TKA without MCL injury. Therefore, repair with a suture anchor is a reliable method that provides good clinical and stability outcomes in patients with MCL injury during TKA.

## 1. Introduction

Ligament balancing is the most crucial part of total knee arthroplasty (TKA). A well-balanced knee is responsible for long term survival of prosthesis. In addition, bony cutting techniques are not universally standardized [1] The most common release during TKA is the release of medial collateral ligament (MCL), particularly in osteoarthritic knees with varus deformity and those with tight medial sleeve and lax lateral structures [2].

The article "Clinical Outcomes of Repair of Complete Detachment of Medial Collateral Ligament at the Tibial Insertion in Bilateral Total Knee Arthroplasty" was published in 2022. Journal: Evid Based Complement Alternat Med.

Subperiosteal elevation of deep and superficial parts of the MCL from the proximal tibia is a commonly used MCL releasing technique. The newer pie crusting technique is usually used in conjunction with the MCL releasing technique [3, 4]. Partial release of the MCL is usually adequate. Although rare, complete detachment of the MCL insertion can occur. It usually occurs in knees needing large correction or in those with obesity [5–7]. Mid-substance injuries to the MCL are rare. They are usually caused by oversized saw blades, intraoperative hyper flexion, or secondary to pie-crusting [6, 8]. Mid-substance tears are managed either by primary repair or augmentation [9]. Avulsions at the femoral or tibial attachment have been treated with various techniques, including screw and washer constructs, suture anchors, and soft tissue staples [10].

Instability resulting from an injury to the MCL is catastrophic, necessitating constrained implants to prevent joint opening upon valgus stress [11, 12]. However, concerns over increased stresses at the implant-cement and cement-bone interface that might cause early loosening have urged surgeons to look for alternatives [10, 13]. Recent studies have shown good results with the use of unconstrained implants in conjunction with primary repair or augmentation [13, 14]. More surprisingly, conservative management by simply upsizing the polyethylene insert has shown good results for the intraoperative detachment of MCL from the tibial attachment site during primary TKA [15, 16]. Being a relatively rare complication (0.7–3% in literature), the detachment of MCL has been studied with moderate size and retrospective nature. To the best of our knowledge, no study has compared outcomes including stability between repaired MCL knee and no injury knee in patients with bilateral TKAs.

Therefore, the purpose of this study was to compare clinical outcomes and stability of repaired knee with complete MCL detachment to those of contralateral knee without MCL detachment in patients with bilateral TKAs. The hypothesis of this study was that the repaired knee with detachment of MCL would be clinically and radiologically equivalent to the contralateral knee without MCL detachment in patients with bilateral TKA.

## 2. Materials and Methods

This was a single tertiary center, retrospective, observational study conducted with the approval of the Institutional Review Board (IRB). Records of 3,365 consecutive primary osteoarthritis (OA) patients (4,417 knees) who received surgery during the period of January 2003 to December 2015 were retrospectively reviewed. Demographic and intraoperative data were gathered from a prospective database maintained at our institute. Among 1,052 patients (2,104 knees) with bilateral TKA, 45 patients (45 knees, 2.1%) had repair for complete MCL detachment at the tibial insertion in one knee (repaired group). MCL in all other contralateral knee was not detached. It was not repaired either (control group). Of 45 patients, two patients had insufficient baseline or postoperative data. Hence, 43 patients were available for analysis after a minimum of 5 years follow-up. They were included in this study (Figure 1).

The article "Clinical Outcomes of Repair of Complete Detachment of Medial Collateral Ligament at the Tibial Insertion in Bilateral Total Knee Arthroplasty" was published in 2022. Journal: Evid Based Complement Alternat Med.

Demographic data including age, gender, and body mass index were collected preoperatively. Clinical outcomes including Knee Society Pain (KSP) score, Knee Society Function (KSF) score, and Western Ontario & McMaster Universities Osteoarthritis (WOMAC) score were compared between the two groups. The active range of motion, maximal flexion, and flexion contracture, if any, were also recorded in the database.

Preoperative and postoperative radiographs available for review included anteroposterior and lateral view, valgus stress views, and weight-bearing full-length teleoroentgenogram. The HKA (Hip-Knee-Ankle) angle were calculated on teleoroentgenograms (Figure 2). Objective quantitative instability was evaluated by measurement of the opening angle in valgus stress radiographs using a Telos device (Telos stress device; Austin & Associates, Fallston, MD, US) under 150 N [5]. Implants of the same design by the same manufacturer were used in both knees of one patient. These implants were posterior-stabilized prostheses, including Vanguard (Zimmer Biomet, Warsaw, IN, USA), NexGen LPS-Flex (Zimmer, Warsaw, IN, USA), Vega (B-Braun, Tuttlingen, GER), and Attune (Depuy, Warsaw, IN, USA). Constrained implants were not used for complete MCL detachment during the study period.

### 2.1. Surgical Procedures

All surgeries were performed by two senior surgeons. Techniques employed were similar throughout the study period. All patients underwent bilateral total knee arthroplasty in the same sitting under combined spinal-epidural or general anesthesia in a supine position with tourniquet inflated. Standard midline medial parapatellar approach was used for all patients. The tibial cut was taken perpendicular to the mechanical axis of tibia with a 3° posterior slope aided by an extramedullary guide. A distal femoral cut was then done using an intramedullary guide with 4–6° of valgus based on anatomical and mechanical axes of the femur. Osteophytes were removed and medial soft tissue release was performed with the aim to achieve a mediolateral balance in extension within 2 mm. The resection line of the posterior femoral cut was drawn on the cut surface of the distal femur parallel to the resected proximal tibia at 90° of knee flexion. Distraction was maintained with a laminar spreader. Posterior and chamfer cutting was then performed after positioning a 4 in 1 cutting block. Stability was checked in 90° of flexion and full extension. The final implant was then cemented. Mediolateral balance was within 2 mm under varus. The valgus stress test was achieved by MCL release. Complete detachment of MCL at tibial attachment was then examined. If there was a presence of the complete detachment of MCL with opening more than 5 mm in extension or at 30° of knee flexion under valgus stress test [9], the site of tibial detachment was fixed with either 5.5 mm suture anchor (Arthrex, Naples, FL, USA) to provide additional stability. Using a free needle, each of the 4 sutures is passed in simple fashion through the substance of the ligament, 2 anteriorly and 2 posteriorly. The proximal anterior and posterior sutures limbs are then tied together with the knee held in 30° of knee.

The article "Clinical Outcomes of Repair of Complete Detachment of Medial Collateral Ligament at the Tibial Insertion in Bilateral Total Knee Arthroplasty" was published in 2022. Journal: Evid Based Complement Alternat Med.

Flexion (Figure 3). After assessing stability and patellar tracking, the surgical wound was closed and surgical drains were put in place in all cases. The contralateral TKA (without complete MCL detachment) was performed in a similar fashion following standard procedure.

Postoperatively, drains were removed at 48 hours and sutures were removed at day 14. MCL repaired knee was protected with a hinged knee brace for 4 weeks. Early, inpatient physiotherapy, and range of motion exercises were initiated for all patients. The protocol was the same for the contralateral without a complete MCL detachment knee, except full weight bearing was delayed for 4 weeks for the complete MCL detachment group.

### 2.2. Statistical Analysis

All data are presented as mean and range standard deviation. Statistical analyses were performed using SPSS statistical software system version 22.0 (IBM Corporation, Armonk, NY, USA). Kolmogorov–Smirnov tests were performed to evaluate whether the data showed a normal distribution or not. For the data with a normal distribution, a Student paired *t*-test was performed to compare outcomes between groups preoperatively, and at the final follow-up, an independent *t*-test was performed for comparison of outcomes between the 2 groups. For the data showing a nonnormal distribution, Mann–Whitney *U* tests were employed for the comparison of outcomes measured preoperatively and at the final follow-up, and between the 2 groups. Statistical significance was set at *p* ≤ 0.05 for all tests. The power analysis determined that a sample of 37 patients in each group was needed to obtain differences of 2° on the change of between the repair and control groups in total stability with a statistical power of 80% and a significance level of 5%.

The article "Clinical Outcomes of Repair of Complete Detachment of Medial Collateral Ligament at the Tibial Insertion in Bilateral Total Knee Arthroplasty" was published in 2022. Journal: Evid Based Complement Alternat Med.

## 3. Results

Of the 43 patients, 41 were females and two were males. Their mean age at surgery was 67 years (range, 59–74 years). The average follow-up duration was 102 months (range, 67–178 months). Their mean body mass index was 27.2 kg/m^2^ (range, 21.1–34.7 kg/m^2^) (Table 1).

The total operative time, blood loss, and insert thickness were not different between the two groups (Table 2).

In the repaired group, the HKA angle was corrected from a mean varus of 11.9° to 0.8° varus after TKA. Similarly, contralateral knee was corrected from a mean varus of 11.2° to 0.8° varus after TKA. Clinically, the range of motion was improved in the repair group from preoperative 117.6° to 125.5° at the final follow-up. The control group also had similar results (from 120.7° preoperatively to 125.6° at the final follow up). Flexion contracture was improved significantly from 8.7° preoperatively to 1.1° at the final follow-up in the repaired group. This was similar to the improvement in the control group (from 7.6° preoperatively to 0.9° at the final follow-up). Differences between the two groups were not statistically significant. There was no significant difference in KSP, KSF, and WOMAC scores between the two groups either preoperatively or at the final follow-up. The stability measured on stress radiographs in extension was 4.1 ± 2.3° in MCL injured and 3.3 ± 2.1° in control groups without statistical significance (*p*=0.208). No significant differences were found on stress radiographs at 30° of knee flexion as well (*p*=0.125). At the final follow-up, no patient complained of knee instability and all patients were capable of community ambulation without any assistive device (Table 3).

## 4. Discussion

The incidence of MCL injury in our series was 2.1%, similar to that in other studies [10, 11]. Similar radiological, clinical, and functional outcomes postoperatively were found for MCL-repaired and MCL nonrepaired knees in the same patient. Although similar studies have been performed in the past, none has compared outcomes of MCL-repaired knees to contralateral uninjured knees after TKA, which can serve as a perfectly matched control group [14, 15].

Collateral ligament injuries can cause coronal plane instability. Constrained implants have long been used as an alternative for treating this problem [17, 18]. Unfortunately, constrained implants are more prone to aseptic loosening due to increased stresses at the implant-cement and the cement-bone interface can also affect the longevity of such implants. Because of these issues, surgeons are considering other alternatives.

The article "Clinical Outcomes of Repair of Complete Detachment of Medial Collateral Ligament at the Tibial Insertion in Bilateral Total Knee Arthroplasty" was published in 2022. Journal: Evid Based Complement Alternat Med.

A Grade III tear to the MCL has propensity to heal spontaneously [19, 20]. Koo and Choi have demonstrated good results in MCL injuries managed conservatively by upsizing polyethylene insert 2-4 mm. However, overstuffing the lateral component, although minimal, might have deleterious long-term effects due to increased PE wear [16].

The PCL is a secondary stabilizer of the knee, counteracting varus, valgus, and rotational stresses encountered by the joint. Previous studies have preferred a cruciate-retaining prosthesis in an MCL-injury scenario [10], evidently taking advantage of the apparent stability provided by the intact PCL [21]. A cruciate-retaining prosthesis might be advantageous if the MCL injury is being managed conservatively. However, primary repair usually bestows some amount of immediate stability to valgus stress, allowing a posterior stabilizing implant to be used. In addition, using a cruciate-retaining prosthesis is difficult for patients with severe varus who are prone to MCL injury as ligament balancing to provide adequate correction is tricky even in the best of hands. Recent studies have used the PS implant successfully [14, 16]. Cho et al. have compared the laxity of MCL-on and MCL-off knees one year postoperatively and found no statistically significant difference. They believe that the implanted prosthesis itself can provide adequate initial stability and allow the MCL to heal [15]. Mukesh et al. found that for MCL injury of proximal or distal side, single-row anchor repairing can achieve good results. This technique reattaches the torn ligament at its near anatomical attachment site using a single, double-loaded 5.5-mm suture anchor [22].

The present study suggests that repair of over-released MCL with suture anchors accompanied by utilization of unconstrained posterior stabilizing prosthesis in primary TKA is an adequate treatment strategy that avoids complications, improves long-term survivorship, and decreases bony resection without a constrained implant.

This study has some limitations. First, this was a retrospective study. Therefore, it might have selection and recall bias. In addition, only one treatment modality was tested, although it provided satisfactory results. It is currently unclear whether constrained prosthesis and conservative approach can provide comparable outcomes.

## 5. Conclusion

For a complete detachment of the medial collateral ligament during total knee arthroplasty, repair with a suture anchor and an unconstrained implant is a reliable treatment method. It provides the clinical and radiological results as good as the total knee arthroplasty without medial collateral ligament injury.

The article "Clinical Outcomes of Repair of Complete Detachment of Medial Collateral Ligament at the Tibial Insertion in Bilateral Total Knee Arthroplasty" was published in 2022. Journal: Evid Based Complement Alternat Med.

## 6. Ethical Approval

The study was approved by our Institutional Review Board (IRB).

## Figures and Tables

**Figure 1:** Flow chart of subjects in the retrospective study.

**Figure 2:** (a) Postoperative teleroentgenography. (b) Valgus stress radiographs of right knee extension; (c) Valgus stress radiographs of left knee extension.

**Figure 3:** (a) Opening in 30° of knee flexion under valgus stress test (b) Detatchment injury of MCL from tibial attachment site; (c) MCL repositioned to tibial site and fixed with suture anchor.

**Table 1:** Demographics of the patients.

Number of patients	43
Gender (Male/Female)	2/41
Age, years (range, SD)	67 (59–74, 7.0)
BMI, kg/m^2^ (range, SD)	27.2 (21.1–34.7, 3.5)
Follow-up time, months (range, SD)	102 (67–178, 33)

SD: standard deviation; BMI:body mass index.

**Table 2:** Comparison of Intraoperative between two groups.

Variable	Repair group	Control group	*p*-value (m)
Total operative time (min)	93.6 ± 20.5	95.3 ± 21.4	0.316
Calculated blood loss (ml)	417.6 ± 176.4	417.7 ± 177.5	0.404
Thickness of insert (mm)	10.4 ± 1.3	10.8 ± 1.9	0.861

^m^Mann–Whitney *U* test.

**Table 3:** Comparison Preoperative and Final follow-up of Clinical results and Stability between two groups.

	Preoperative			Final follow-up		
	Repair group	Control group	*p*-value	Repair group	Control group	*p*-value
HKA angle (degree)	−11.9 ± 4.1	−11.2 ± 4.4	0.522^m^	−0.8 ± 1.7	−0.8 ± 2.6	0.967^m^
Range of motion (degree)	117.6 ± 17.4	120.7 ± 13.5	0.404^m^	125.5 ± 10.9	125.6 ± 7.5	0.381^m^
Maximum flexion (degree)	126.4 ± 14.3	128.4 ± 10.4	0.461^m^	126.7 ± 8.7	126.5 ± 6.9	0.344^m^
Flexion contracture (degree)	8.7 ± 7.1	7.6 ± 7.2	0.535^m^	1.1 ± 2.8	0.9 ± 2.3	0.691^m^
KS pain (points)	23.5 ± 11.3	27.1 ± 12.2	0.067^m^	45.8 ± 4.2	44.9 ± 5.4	0.242^m^
KS function (points)	45.3 ± 14.2	51.8 ± 11.6	0.088^s^	86.3 ± 8.1	88.1 ± 9.6	0.692^s^
WOMAC (points)	69.9 ± 13.9	64.8 ± 10.9	0.124^s^	19.1 ± 8.9	17.6 ± 10.1	0.546^m^
Stability (degree)						
Extension	2.2 ± 2.8	2.1 ± 3.1	0.718^s^	4.1 ± 2.3	3.3 ± 2.1	0.208^m^
30°Flexion	2.6 ± 3.2	3.6 ± 3.7	0.072^s^	5.9 ± 2.6	4.9 ± 2.7	0.125^m^

HKA: Hip-Knee-Ankle (-:varus); KS: Knee Society; WOMAC:Western Ontario and McMaster University Osteoarthritis Index. Stability: Measurements of medial opening angles on valgus stress. ^s^Student paired *t*-test; ^m^Mann–Whitney *U* test.

## Data Availability

In this retrospective analytical study, data were collected from Chonnam National University Hwasun Hospital digital medical registry.
